The article "Evaluating the Effect of QIIME Balanced Default Parameters on Metataxonomic Analysis Workflows With a Mock Community" was published in 2019. Journal: Front Microbiol.

# Evaluating the Effect of QIIME Balanced Default Parameters on Metataxonomic Analysis Workflows With a Mock Community

**DOI:** 10.3389/fmicb.2019.01084

**Published:** 2019-05-16

**Authors:** Dimitrios Kioroglou, Albert Mas, Maria del Carmen Portillo

**Affiliations:** Department Biochemistry and Biotechnology, Faculty of Oenology, University Rovira i Virgili, Tarragona, Spain

**Keywords:** metataxonomics, next-generation-sequencing, bioinformatics, QIIME, PCR, Ion Torrent, Illumina, wine

## Abstract

Metataxonomic analysis represents a fast and cost-effective approach for acquiring informative insight into the composition of the microbiome of samples with variable diversity, such as wine samples. Nevertheless, it comprises a vast amount of laboratory procedures and bioinformatic frameworks each one associated with an inherent variability of protocols and algorithms, respectively. As a solution to the bioinformatic maze, QIIME bioinformatic framework has incorporated benchmarked, and balanced parameters as default parameters. In the current study, metataxonomic analysis of two types of mock community standards with the same microbial composition has been performed for evaluating the effectivess of QIIME balanced default parameters on a variety of aspects related to different laboratory and bioinformatic workflows. These aspects concern NGS platforms, PCR protocols, bioinformatic pipelines, and taxonomic classification algorithms. Several qualitative performance expectations have been the outcome of the analysis, rendering the mock community a useful evaluation tool.

## 1. Introduction

During the past years significant improvements in Next Generation Sequencing (NGS) platforms and computational performance have given a considerable momentum to the research of microbial communities. Primarily there are two sequencing-based methods for the classification analysis of a microbiome, the metagenomic approach which concerns the shotgun sequencing of microbial DNA, and the metataxonomic approach which refers to the sequencing of a marker gene, having as a usual target the ribosomal RNA gene (Breitwieser et al., 2017). Due to the cost-effectiveness and decreased demands on computational resources of the latter, it has been used quite broadly in research and consists the focus of the current study.

A typical metataxonomic analysis includes a process that combines laboratory and bioinformatic workflows. The steps involved in the laboratory process concern the collection of a microbiome sample, the DNA extraction, the library preparation based on the preferred rRNA gene marker and the massive sequencing with the NGS platform of choice. The bioinformatic workflow concerns the quality filtering of the resulted data, the clustering of sequences based on a specific clustering strategy and the taxonomic assignment to the representative sequence of each cluster.

The article "Evaluating the Effect of QIIME Balanced Default Parameters on Metataxonomic Analysis Workflows With a Mock Community" was published in 2019. Journal: Front Microbiol.

There are a plethora of bioinformatic frameworks for the analysis of the microbiome data with Quantitative Insights Into Microbial Ecology (QIIME) being one of the most popular and thus, implemented in the current study (Caporaso et al., 2010; Bolyen et al., 2018). As a bioinformatic framework, it contains a significant amount of algorithms and parameters to select and tweak, respectively, but studies such as Bokulich et al. (2013, 2018) have provided informative and useful benchmarks with the resulted balanced parameters being incorporated into QIIME as default parameters. Nevertheless, microbiome samples are subjects to different laboratory procedures and protocols and as such implementation of parameters must be evaluated. For that reason, a mock community, which represents a microbiome sample of known composition (Bokulich et al., 2016), consists a valuable tool in assessing both laboratory and bioinformatic workflows prior to establishment of parameters. There are many studies dedicated to mock communities, such as Yuan et al. (2012) where a mock community was used for the comparison of six common DNA extraction protocols, or Yeh et al. (2018) where mock communities were the tool for the establishment of a methodology that could verify similar performance between sequencing runs. However, the way that the current study differs from the rest is based on the fact that the main focus is given on assessing the effectiveness of QIIME balanced default parameters on our laboratory and bioinformatic workflows destined to the metataxonomic analysis of wine samples.

Wine samples are characterized by extremely dynamic microbial populations. During wine ageing, these populations tend to be quite sparse with most of the microorganisms being difficult to detect as they enter the viable but non-culturable state (VBNC) (Millet and Lonvaud-Funel, 2000), and thus making NGS technology the most appropriate detection tool. Therefore, sparse microbial communities are quite important since wine spoilage microorganisms may go undetected due to their low abundance and significantly alter the wine quality later on. For that reason, the mock community in the current study was chosen to be simple. Additionally to the main focus, the mock community will serve a double qualitative role on a series of aspects related to our workflows. Regarding the laboratory procedure, to evaluate 16S metataxonomic analysis on data produced by Ion Torrent and Illumina platforms, the impact of 18S and ITS amplicons on the metataxonomic classification and the effect of the PCR cycles during the library preparation on the downstream bioinformatic analysis of the Ion Torrent data. As far as the bioinformatic analysis is concerned, the mock community will assist in ascertaining the impact on classification of different quality filtering thresholds, the performance of different sequence clustering methods and the classification performance of two different algorithms. Moreover, we are examining the possibility of utilizing the confidence of the assigned taxonomy, as reported by the classification algorithms, as a tool for eliminating false positives.

The article "Evaluating the Effect of QIIME Balanced Default Parameters on Metataxonomic Analysis Workflows With a Mock Community" was published in 2019. Journal: Front Microbiol.

## 2. Methods

### 2.1. Laboratory Workflow

Two microbial community standards from ZymoBIOMICS^*TM*^ with the same microbial composition of 8 prokaryotes and 2 eukaryotes and impurity level < 0.01% have been used. The first standard contained DNA extracted from pure cultures (DNA standard D6305 200 ng), whereas the second standard was constructed by pooling pure cultures (Microbial Community standard D6300). The microbial species along with the 16S theoretical relative abundance, as provided by the standards specifications, are given in Table 1. The theoretical relative abundances have been calculated by the standards provider taking into consideration differences in the number of copies each amplicon has among the species. However, such correction is rendered impossible when estimating relative abundances in real wine samples. Therefore, the estimated relative abundances have not been corrected in order to examine the amount of deviation between estimated and ideal relative abundance. The aim of using the DNA standard (DS) was to assess the performance of different PCR primers and amplicons used with the NGS platforms, the impact of PCR cycles on the number of chimeric sequences in the Ion Torrent platform, as well as the performance of the bioinformatic pipelines at reconstructing the 16S theoretical relative abundance as well as assigning correct taxonomy to the eukaryotic DNA. The additional goal of using the culture standard (CS) was to ascertain the effectiveness of the in-house DNA extraction protocol that follows the recommended procedure of the DNeasy Plant Mini kit (Qiagen, Hilden, Germany), including three bead-beating steps for 3 minutes in a FastPrep-24 bead beater (MP Bio, Solon, OH) (Lleixà et al., 2018).

**Table 1:** Culture and DNA standard microbial composition of the mock communities used during the current study and 16S theoretical relative abundance.

**Species**	**NRRL accession NO**.	**Theoretical composition of 16S rRNA(%)**	
		**Culture standard**	**DNA standard**
*Pseudomonas aeruginosa*	B-3509	4.2	4.6
*Escherichia coli*	B-1109	10.1	10.0
*Salmonella enterica*	B-4212	10.4	11.3
*Lactobacillus fermentum*	B-1840	18.4	18.8
*Enterococcus faecalis*	B-537	9.9	10.4
*Staphylococcus aureus*	B-41012	15.5	13.3
*Listeria monocytogenes*	B-33116	14.1	15.9
*Bacillus subtilis*	B-354	17.4	15.7
*Saccharomyces cerevisiae*	Y-567	-	-
*Cryptococcus neoformans*	Y-2534	-	-

*Based on ZymoBIOMICS^TM^, the strain information was extracted from the website of the Agricultural Research Service Culture Collection and can be accessed with the NRRL accession number (NRRL, https://nrrl.ncaur.usda.gov/)*.

The article "Evaluating the Effect of QIIME Balanced Default Parameters on Metataxonomic Analysis Workflows With a Mock Community" was published in 2019. Journal: Front Microbiol.

Amplicon based sequences were generated by two different platforms, Ion Torrent (Centre for Omics Sciences, Reus, Spain) and Illumina (Centre for Genomic regulation, Barcelona, Spain). In the case of Ion Torrent, the sequencing libraries were prepared in the in-house laboratory of the University Rovira i Virgili using both the DNA and culture standard. For the libraries creation, the 16S rRNA region was amplified by PCR with the primers 515F and 806R (Caporaso et al., 2011) whereas the 18S rRNA region was amplified using the primers FR1 and FF390 (Prevost-Boure et al., 2011). Since a positive correlation between PCR cycles and amount of chimeric sequences has been reported (Ahn et al., 2012), 30 and 45 PCR cycles were used for the libraries creation. The PCR products were purified using GeneRed Size selection Kit (Qiagen, Hilden, Germany) and sent to COS for sequencing with the 530 chip using the Gene Studio S5 System of the Ion Torrent platform. On the other side, the DNA standard and extracted DNA from the culture standard were sent directly to CRG to be sequenced by Illumina MiSeq 2x300 yielding paired end sequences for the v3 region of the 16S [primers 341F and 785R, Herlemann et al. (2011)] and for the ITS region [primers ITS1F/ITS2R, White et al. (1990)]. Schematic representation of the experimental design is given in Figure 1.

**Figure 1:** Two commercial mock community standards from ZymoBIOMICS™ with exactly the same microbial composition of 8 prokaryotes and 2 eukaryotes have been used in the current study. The Microbial Community standard (referred as CS) consisted of microbial cells from which DNA was extracted using an in-house DNA extraction protocol. The DNA standard (referred as DS) contained DNA from the same 10 microbial cells as the CS but extracted by ZymoBIOMICS™. Both standards were sequenced using Ion Torrent and Illumina platforms. Regarding the DNA from the prokaryotic cells, both platforms sequenced the 16S amplicon. Regarding the DNA from the eukaryotic cells, Ion Torrent sequenced the 18S amplicon whereas Illumina the ITS amplicon. In the case of Ion Torrent 30 and 45 PCR cycles have been implemented in both amplicons, whereas in Illumina only 30 PCR cycles were implemented. Sequencing data derived from both NGS platforms have been analyzed using QIIME 1 and QIIME 2.

The article "Evaluating the Effect of QIIME Balanced Default Parameters on Metataxonomic Analysis Workflows With a Mock Community" was published in 2019. Journal: Front Microbiol.

The Ion Torrent platform generated in average 300 bp reads for the 16S amplicon and 350 bp reads for the 18S amplicon, with an average Phred33 quality score of 29 and 27, respectively. On the other hand, Illumina generated in average 300 bp reads for both amplicons with an average Phred33 quality score of 36 for both 16S and ITS forward reads and 34 and 35 for the 16S and ITS reverse reads, respectively. Due to the fact that the Phred33 quality of the Ion Torrent reads dropped below 10 in positions located in the middle of the read, two filtering strategies were applied. One applying a quality threshold at 10 (Q10) and one at 20 (Q20). The motivation behind these two strategies was to examine whether higher number of sequences or higher overall quality will produce better results. Contrarily, for the Illumina reads, only the Q20 threshold was applied.

### 2.2. Bioinformatic Workflow

Bokulich et al. (2013) benchmarked different quality filtering strategies with QIIME 1 and Bokulich et al. (2018) benchmarked the performance of difference classification algorithms between QIIME 1 and QIIME 2. Therefore, the bioinformatic pipelines were based on two versions of QIIME, QIIME 1 (version 1.9.1) and QIIME 2 (version 2018.2), with the processing and taxonomic assignment steps mentioned in Table 2. Along with QIIME, bioinformatic tools such as FastQC (Andrews, 2010), Trimmomatic (Bolger et al., 2014) and FLASH (Magoč and Salzberg, 2011) were executed externally.

**Table 2:** Bioinformatic pipelines based on NGS platform and method of clustering used during this study for comparison of their performance over the mock community standards.

**Ion Torrent OTU**	**Illumina OTU**	**Illumina ASV**
Barcode extraction*^a^*	Paired ends merging*^c^*	Paired ends merging*^c^*
Quality filtering (Q10 or Q20)*^a^*	Quality filtering (Q20)*^d^*	DADA2 quality filtering (Q20)*^b^*
Reads dereplication*^b^*	Reads dereplication*^b^*	DADA2 reads dereplication*^b^*
Open reference OTU*^b^*	Open reference OTU*^b^*	DADA2 Chimeras filtering (only ITS)*^b^*
Chimeras filtering*^b^*	Chimeras filtering*^b^*	DADA2 ASV*^b^*
SKLEARN classifier training*^b^*	SKLEARN classifier training*^b^*	SKLEARN classifier training*^b^*
SKLEARN taxonomy assignment*^b^*	SKLEARN taxonomy assignment*^b^*	SKLEARN taxonomy assignment*^b^*
BLAST+ taxonomy assignment*^b^*	BLAST+ taxonomy assignment*^b^*	BLAST+ taxonomy assignment*^b^*

a *QIIME 1 ( version 1.9.1 )*.

b *QIIME 2 ( version 2018.2 )*.

c *FLASH*.

d *Trimmomatic*.

The article "Evaluating the Effect of QIIME Balanced Default Parameters on Metataxonomic Analysis Workflows With a Mock Community" was published in 2019. Journal: Front Microbiol.

From the default parameters of QIIME 1 for the quality filtering of raws reads, only the Phred33 quality threshold was altered. Generally, the quality filtering concerned discarding reads with consecutive bases above a given Phred33 threshold but occupying < 75% of the total read length, truncating reads at positions with more than 3 consecutive bases with Phred33 quality less than the desired and reassessing the discarding rule after truncation. Due to the fact that QIIME 1 quality filtering steps require the sequences to be multiplexed, for the demultiplexed Illumina sequences the quality filtering steps of QIIME 1 were replicated in Trimmomatic. Moreover, the DADA2 algorithm (Callahan et al., 2016), as incorporated into QIIME, truncated reads at the first base instance of undesired quality and discarded reads with >2 expected errors. An additional filtering step was implemented by removing chimeric sequences with VSEARCH UCHIME de novo (Rognes et al., 2016) or DADA2.

Regarding the Illumina reads two clustering methods were applied. One that creates clusters of sequences, called operational taxonomic units (OTU) based on a similarity threshold (Rideout et al., 2014) and one that defines sequence variants called amplicon sequence variants (ASV) (Callahan et al., 2017). The OTU method produces an OTU-table where, for each sample, the number of sequences in each OTU has been recorded (Rognes et al., 2016), whereas the ASV method is related with an ASV-table of the frequency that each ASV has been observed in each sample (Callahan et al., 2016). OTUs containing < 10 sequences across all samples were filtered-out as noise (Giordano et al., 2018), and the similarity threshold for the OTU clustering was set to 99% as this threshold returns more comparable results between OTU and ASV (Van Der Pol et al., 2018).

For the metataxonomic classification the database SILVA (version 132) has been the source of taxonomy for the 16S and 18S amplicons (Quast et al., 2012) as it is the most recent and updated database, whereas the ITS taxonomy relied on the UNITE database (version 7.2) (Nilsson et al., 2018). The taxonomic assignment was carried out by two algorithms, the k-mer based multinomial naive Bayes algorithm integrated in the Python Scikit-learn library (SKLEARN) (Pedregosa et al., 2011) and the Basic Local Alignment Search Tool+ (BLAST+) algorithm which represents an enhanced version of the very popular BLAST algorithm available from 1997 (Camacho et al., 2009). Both algorithms report a confidence percentage, with the SKLEARN algorithm referring to the amount of confidence for the taxonomy assigned at a specific taxonomic level and BLAST+ referring to the fraction of top hits that matched the consensus taxonomy at a given level. As SKLEARN represents a machine learning approach, the additional flexibility provided was to assign taxonomy after training the algorithm with extracted reference sequences from the SILVA and UNITE databases using the aforementioned PCR primers and trimmed to a length equal to the maximum length of the reads after quality filtering. The training process of SKLEARN is based on k-mers where the value 7 was used as it is the default balanced QIIME 2 parameter. In relaxed terms, during the training process SKLEARN splits each reference sequence into a series of overlapping heptamers and assigns a level of taxonomy to a given collection of heptamers. Later on, during the classification process SKLEARN splits each sequence once again into a collection of overlapping heptamers, and tries to assign a level of taxonomy by taking into consideration the collections of heptamers from the reference sequences. The balanced default parameters of BLAST+ remained unaltered whereas the performance of SKLEARN improved after reducing the confidence parameter from the default 0.7 value down to 0.5.

The article "Evaluating the Effect of QIIME Balanced Default Parameters on Metataxonomic Analysis Workflows With a Mock Community" was published in 2019. Journal: Front Microbiol.

## 3. Results

Figure 2 shows the number of sequences for each sample after applying Phred33 quality filtering and removing chimeras. For the Ion Torrent a mild filtering was applied after setting the quality threshold at Q10 with an average of 8.6% of the sequences filtered, across all samples, for the 16S amplicon and 14.1% for the 18S whereas at Q20 an average of 62 and 72.4% was removed, respectively. An additional average of 13.5% of the sequences were identified as chimeras for the 16S amplicon and 1.2% for the 18S at Q10, while at Q20 the identified chimeras were 5.9 and 1.3%, respectively. Considering the PCR cycles, their impact on the production of chimeras was not clear for the 16S amplicon as at Q10, 45 cycles generated 3.5% more chimeras than 30 cycles for the CS but for the DS they produced 4.2% less. The same pattern repeated for the 16S amplicon at Q20 with 45 cycles of the CS producing 1.6% more chimeras but for the DS 3.5% more chimeras produced from 30 cycles. On the other hand, the difference was more apparent for the 18S amplicon producing more chimeras at 45 than 30 cycles, but the difference was marginal representing only 1.6% of the sequences in average (Figure 2A).

**Figure 2:** Number of sequences resulted after applying quality and chimeras filtering. **(A)** Ion Torrent. First letter of the sample names (C or D) represents type of mock community standard (Culture or DNA). What follows is the number of PCR cycles (30 or 45) with the amplicon (16S or 18S) at the end. The raw number of sequences are represented in green and in red and blue the two Phred33 quality filtering strategies Q20 and Q10, respectively. **(B)** Illumina. First letter of the sample names (C or D) represents type of mock community standard (Culture or DNA) with the amplicon (16S or ITS) at the end. The raw number of sequences are represented in green and in red and blue the sequences resulted from the filtering steps of the Illumina ASV and Illumina OTU pipeline, respectively.

The article "Evaluating the Effect of QIIME Balanced Default Parameters on Metataxonomic Analysis Workflows With a Mock Community" was published in 2019. Journal: Front Microbiol.

For the Illumina platform, the merging of the paired ends caused a ≈2% loss of reads for the 16S amplicon in both standards, whereas for the ITS amplicon of the DS the loss was 38%. Due to the fact that the sequencing of the ITS amplicon for the CS generated very low amount of sequences which had very low Phred33 quality, this sample was excluded from the study. This was the additional reason for not reporting the theoretical abundance of 18S and ITS amplicons, along with the fact that from the two standards only the CS reports 18S theoretical abundance in the specifications. However, research interest still remained on examining whether the classification algorithms could assign correct taxonomy to the eukaryotic DNA and which amplicon of the two improves classification performance. For the 16S amplicon of the CS, the Illumina OTU pipeline removed 1.2% of sequences during the quality filtering step and an additional 23.7% was identified as chimeras. The pipeline performed quite similar for the DS removing 1 and 17.9%, respectively. On the contrary, for the 16S amplicon of the two standards the Illumina ASV pipeline identified ≈80% of the sequences as chimeric. This high percentage could be justified in cases where non-biological nucleotides, such as primers or adapters, have not been removed prior to analysis ^1^, but since this rationale did not hold for the given dataset, the chimera filtering step was omitted for both standards. Therefore, the only loss was during the quality filtering with both standards losing ≈5% of sequences. Regarding the ITS amplicon of the DS, the Illumina OTU pipeline filtered 0.8% of sequences based on quality but did not identify any chimeras, and the Illumina ASV pipeline removed 1.9% during quality filtering and a further 5% during chimera filtering (Figure 2B).

The metataxonomic classification was performed at genus level since accurate classification at species level is a known limitation of rRNA amplicon sequencing due to the fact that it is a highly conserved region (Sentausa and Fournier, 2013). This limitation became apparent also in the current study as the only bacterium identified consistently and accurately at species level was *Listeria monocytogenes* whereas *Salmonella* was the only one whose classification never reached species level. From the rest, *Bacillus* demonstrated the highest variability with overall 7 different species being identified, 5 species for *Staphylococcus* and *Pseudomonas*, and ≤ 3 for *Escherichia, Lactobacillus*, and *Enterococcus*. Although this broad variability concerned the OTU clustering method, the variability in the ASV method was more constrained including only the cases of either correct species identification, no species identification or species identification as *uncultured bacterium*.

The article "Evaluating the Effect of QIIME Balanced Default Parameters on Metataxonomic Analysis Workflows With a Mock Community" was published in 2019. Journal: Front Microbiol.

Figures 3–**6** depict 16S estimated relative abundance (orange color) being juxtaposed against theoretical relative abundance (blue color) for both standards and NGS platforms. Overlapping between the two abundances is being represented with dark gray color and estimated abundance below 1% or undefined (0%) is being represented numerically. Excess of orange color at the bar edges denotes abundance overestimation whereas excess of blue color abundance underestimation. Next to each figure the taxonomic assignment confidence is being displayed as it has been reported by the classification algorithm at genus level (All). An additional step has been performed where the assigned taxonomies have been filtered by setting a confidence threshold which is displayed next to the unfiltered confidence. This threshold was initially set to 90% (>0.90) and gradually decreased until an optimal balance between amount of false positives and theoretical abundance reconstruction is achieved. Apart from **Figures 5B**, **6B,D** this confidence threshold matches the minimum unfiltered confidence reported by the classification algorithm giving an identical estimated relative abundance before and after confidence filtering as well as the same amount of false positives (FP).

**Figure 3:** 16S theoretical (blue color) and estimated (orange color) relative abundance for culture standard using Ion Torrent. Overlapping between the two abundances is being represented with dark gray color. Cult_30 and Cult_45 represent 30 and 45 PCR cycles, Q10, and Q20 Phred33 quality filtering threshold and FP false positives without (first number) and with confidence filtering (second number). Figures to the left **(A,C,E,G)** represent estimated abundance based on SKLEARN algorithm and to the right **(B,D,F,H)** based on BLAST+. Estimated relative abundance to the left side of 0 is based on unfiltered confidence (All) and to the right on filtered (> %).

For the Ion Torrent platform, SKLEARN failed to identify *Salmonella* regardless quality filtering threshold, PCR cycles or standard type, while achieved best performance with the DS, 45 PCR cycles, Q20 and confidence threshold 80% (Figure 4G). Overall, the maximum number of false positives was 2 with the genera *Carnobacterium, Citrobacter, Oenococcus*, and *Pediococcus* consisting the pool of false positives. At the same time, BLAST+ seems to have exhibited a better performance than SKLEARN with optimal performance also with the DS, 45 cycles and Q20 (Figure 4H), but generating higher amounts of false positives and requiring a lower confidence threshold for optimal performance. In general, BLAST+ proved to be more sensitive than SKLEARN with 5 as the maximum number of false positives and a persistent confidence threshold of 60%. The false positives identified by BLAST+ were the genera *Cedecea, Citrobacter, Enterobacter, Klebsiella, Oenococcus*, and *Pediococcus*.

The article "Evaluating the Effect of QIIME Balanced Default Parameters on Metataxonomic Analysis Workflows With a Mock Community" was published in 2019. Journal: Front Microbiol.

**Figure 4:** 16S theoretical (blue color) and estimated (orange color) relative abundance for DNA standard using Ion Torrent. Overlapping between the two abundances is being represented with dark gray color. DNA_30 and DNA_45 represent 30 and 45 PCR cycles, Q10, and Q20 Phred33 quality filtering threshold and FP false positives without (first number) and with confidence filtering (second number). Figures to the left **(A,C,E,G)** represent estimated abundance based on SKLEARN algorithm and to the right **(B,D,F,H)** based on BLAST+. Estimated relative abundance to the left side of 0 is based on unfiltered confidence (All) and to the right on filtered (> %).

With Illumina generated data, the landscape was more clear. Both pipelines, Illumina OTU and ASV, yielded similar results with both classification algorithms performing better with the DS (Figure 6). Once again BLAST+ held the best performance managing to approximate quite accurately the theoretical composition (Figures 6B,D). However, it demonstrated overall higher sensitivity producing more false positives with their number being affected by even a slight increase of the confidence threshold by just 1% from the minimum reported confidence of 69% (Figures 5B, 6B,D). The pool of false positives for SKLEARN was comprising the genera *Acetobacter, Enterobacter*, and *Oenococcus*, whereas for BLAST+ the genera *Citrobacter, Acetobacter, Cronobacter, Enterobacter*, and *Oenococcus*. In general, although the relative abundance of the false positives remained below 0.01%, the only excemption was with the CS and the Illumina ASV pipeline where *Cronobacter* reached 0.3%. Moreover, even if the confidence level of the classification assignment was quite low for the false positives in both algorithms (60%), the genera that defied this trend were *Acetobacter, Enterobacter* and *Oenococcus* reaching as high as 90% confidence.

The article "Evaluating the Effect of QIIME Balanced Default Parameters on Metataxonomic Analysis Workflows With a Mock Community" was published in 2019. Journal: Front Microbiol.

**Figure 5:** 16S theoretical (blue color) and estimated (orange color) relative abundance for culture standard using Illumina. Overlapping between the two abundances is being represented with dark gray color. OTU and ASV represent Illumina OTU and Illumina ASV pipelines and FP false positives without (first number) and with confidence filtering (second number). Figures to the left **(A,C)** represent estimated abundance based on SKLEARN algorithm and to the right **(B,D)** based on BLAST+. Estimated relative abundance to the left side of 0 is based on unfiltered confidence (All) and to the right on filtered (> %).

**Figure 6:** 16S theoretical (blue color) and estimated (orange color) relative abundance for DNA standard using Illumina. Overlapping between the two abundances is being represented with dark gray color. OTU and ASV represent Illumina OTU and Illumina ASV pipelines and FP false positives without (first number) and with confidence filtering (second number). Figures to the left **(A,C)** represent estimated abundance based on SKLEARN algorithm and to the right **(B,D)** based on BLAST+. Estimated relative abundance to the left side of 0 is based on unfiltered confidence (All) and to the right on filtered (> %).

With respect to fungi, none of the algorithms detected *Cryptococcus* regardless NGS platform or standard type, contrary to *Saccharomyces* which was detected though not always at species level. In both Illumina OTU and ASV pipelines, both algorithms exhibited similar performance by identifying only *Saccharomyces* with 100% confidence without yielding any false positives. On the other hand, BLAST+ in Ion Torrent managed to identify *Saccharomyces* with 99.9% confidence in both standards regardless quality threshold and PCR cycles, but produced *Zygosaccharomyces* as a false positive with CS at Q10 and 30 cycles and *Kazachstania* with DS at Q20 and 45 cycles having a 60% confidence in both cases. On the side of SKLEARN, *Saccharomyces* occupied ≈61% of the relative abundance in average across the different PCR cycles in both standards at Q10 with the rest of the abundance being occupied by a taxonomy assigned as *uncultured fungus*. At Q20, *Saccharomyces* occupied 99% of the relative abundance with the DS at 45 cycles and 50% in the rest of the samples, with the remaining abundance once again assigned as *uncultured fungus*. Although in the case of BLAST+ the false positives could be removed by raising the confidence threshold, in the case of SKLEARN confidence filtering did not improve the result as the confidence level was in average 90% for *Sacchraromyces* and 85% for the false positives.

The article "Evaluating the Effect of QIIME Balanced Default Parameters on Metataxonomic Analysis Workflows With a Mock Community" was published in 2019. Journal: Front Microbiol.

## 4. Discussion

A mock community represents a microbiome sample of known microbial composition and in the current study two types of mock community standards with the same species composition have become the tool for evaluating the effectiveness of QIIME balanced default parameters on metataxonomic analysis workflows destined to the analysis of wine aging samples. The evaluation was performed with QIIME framework and two classification algorithms, one representing a popular local alignment algorithm (BLAST+) and the other one a popular machine learning approach (SKLEARN). These two algorithms have been introduced for the first time in QIIME 2 and their performance compared to the classification algorithms of QIIME 1 have been benchmarked by Bokulich et al. (2018) where they exhibited similar as well as enhanced performance on different performance metrics. Moreover, Bokulich et al. (2013) in QIIME 1 benchmarked different quality-filtering strategies so as to provide guidelines for processing Illumina amplicon-based sequencing data. Although the suggested parameters of these studies have been incorporated as balanced default parameters in QIIME, microbiome samples undergo different laboratory procedures and protocols and thus these parameters should be evaluated prior to implementation. Therefore, the aim of the present study was to examine the effect of these parameters on a series of aspects related to our laboratory and bioinformatic workflows using a mock community and focusing on reconstructing the theoretical 16S relative abundance or yeast composition based on 18S and ITS amplicon sequencing. Furthermore, the mock community facilitated the qualitative assessment of other aspects such as the performance of the classification algorithms, the possibility of utilizing the reported taxonomic assignment confidence from the classification algorithms as a tool for eliminating false positives, the performance of Ion Torrent and Illumina NGS platforms with the 16S amplicon, the effect of PCR cycles on the analysis of Ion Torrent data, as well as the outcome of the in-house DNA extraction protocol by using a culture based standard (CS).

The 16S metataxonomic analysis of the CS approximated quite closely the outcome of the DS analysis in the Illumina platform, while it demonstrated an apparent variability in the case of the Ion Torrent platform. On the other hand, the Ion Torrent 18S analysis produced similar results in both standards. This denotes that pinpointing a performance culprit among the NGS platforms, PCR protocols or bioinformatic pipelines is rendered difficult as a further variability is being added by the DNA extraction protocol. Regarding the discard of the ITS amplicon based sample of the CS due to low quality, it has been attributed to the poor performance of the DNA extraction protocol since good quality Illumina sequences were generated with the corresponding sample of the DS.

The article "Evaluating the Effect of QIIME Balanced Default Parameters on Metataxonomic Analysis Workflows With a Mock Community" was published in 2019. Journal: Front Microbiol.

With Ion Torrent, both classification algorithms performed better with the DS linked to 45 PCR cycles and Q20 as a quality threshold signifying that optimal performance is more related to better overall sequence quality rather than higher amount of sequences as produced by the Q10 threshold. This could be associated with the fact that Q20 is related to 1% base call error rate while Q10 to 10% (Ewing and Green, 1998), indicating that low Phred33 quality threshold might lead to higher possibility of misclassification. Nevertheless, this result could not be easily attributed to the PCR cycles as 45 cycles in DS produced the highest amount of sequences among all samples and on the other hand in CS both algorithms favored 30 cycles. Moreover, the impact of PCR cycles on the amount of chimeric sequences was either marginal or unclear, however a negative correlation between quality threshold and amount of chimeras became apparent with the 16S amplicon, with fewer chimeras being identified at Q20 threshold. This indicates that a small increase of the PCR cycles does not influence greatly the production of chimeras and many of those chimeric sequences had overall low quality as they represent PCR artifacts. Similarly, slight difference on the production of chimeric sequences was also observed by a small increase of PCR cycles in the study of Ahn et al. (2012) when 25 PCR cycles were compared to 30 cycles, however great disparity on the amount of chimeras was observed between 15 and 30 cycles with the authors suggesting the lowest PCR cycles possible.

As Van Der Pol et al. (2018) suggested, setting the similarity threshold to 99% for the OTU clustering method produced similar results as the ASV method in Illumina, however the latter demonstrated a narrower variability of taxonomic assignment at species level. Furthermore, the omitted chimera filtering step in Illumina ASV pipeline for the 16S amplicon highlighted its importance as false positives above the impurity level of 0.01% were emerged. Additionally, the two NGS platforms presented different filtering behaviors at Q20 with Ion Torrent removing more sequences during the Phred33 quality filtering and less during chimera filtering, whereas Illumina performed the opposite. That could indicate that more chimeric sequences with high Phred33 quality score were generated with Illumina.

As a whole, BLAST+ exhibited better and more balanced performance in both NGS platforms than SKLEARN, however it demonstrated higher sensitivity producing more false positives and overall lower confidence regarding taxonomic assignment. The low amount of false positives generated by SKLEARN with the 16S amplicon could be associated with its training process as higher amount of reference sequences were extracted from the database with the PCR primers of this amplicon compared to 18S and ITS. Nonetheless, its enhanced performance with the Illumina data could be connected to the fact that its default parameters were linked with this NGS platform in the study of Bokulich et al. (2018). Moreover, the lack of false positives from both algorithms with the ITS amplicon could be explained by its higher specificity compared to 18S (Trtkova and Raclavsky, 2006), and overall the reported taxonomic assignment confidence from the algorithms could not lead to an effective filtering tool of false positives as some of the false taxonomies have been assigned with high confidence level.

The article "Evaluating the Effect of QIIME Balanced Default Parameters on Metataxonomic Analysis Workflows With a Mock Community" was published in 2019. Journal: Front Microbiol.

## 5. Conclusions

Overall, the mock community standards have been proven a useful tool demonstrating good performance of QIIME balanced default parameters on our workflows especially with the Illumina platform. Nevertheless, the performance of the NGS platforms or the classification algorithms should not be considered deterministic since an exhaustive benchmarking process is needed for that purpose. As underlined by Bokulich et al. (2018), further fine-tuning of the QIIME default parameters with limited number of mock communities could lead closer to an overfitted rather than generalized performance. Moreover, a series of qualitative performance expectations could be proposed that could be summarized as better metataxonomic outcome when setting the Phred33 quality filtering threshold as high as possible, marginal difference in chimeras production between 30 and 45 PCR cycles, less false positives with ITS amplicon sequencing compared to 18S, similar performance between ASV and OTU clustering method when the clustering similarity threshold of the latter is set to 99% and more comparable results between Ion Torrent and Illumina platforms using the BLAST+ classification algorithm.

## Data Availability

All raw sequencing data used in the current study have been deposited into Sequence Read Archive (SRA) repository under the BioProject accession number PRJNA524645. The raw data are publicly available from the NCBI BioProject database (https://www.ncbi.nlm.nih.gov/bioproject/).

## Author Contributions

AM and MP contributed to the experimental design, funding of the study and writing of the discussion section of the paper. DK performed the DNA extraction, bioinformatic analysis, and writing of the paper. However, all authors had a substantial, direct, and equal intellectual contribution to this study.

The article "Evaluating the Effect of QIIME Balanced Default Parameters on Metataxonomic Analysis Workflows With a Mock Community" was published in 2019. Journal: Front Microbiol.

### Conflict of Interest Statement

The authors declare that the research was conducted in the absence of any commercial or financial relationships that could be construed as a potential conflict of interest.

## Footnotes

^1^https://benjjneb.github.io/dada2/tutorial.html
